The article "Analysis of HFE impact of COVID-19 on OHS in construction enterprises" was retracted in 2025. Reason: concerns about the citations.

# Analysis of HFE impact of COVID-19 on OHS in construction enterprises

**DOI:** 10.1016/j.heliyon.2024.e41275

**Published:** 2024-12-16

**Authors:** Zhonghong Cao, Junjie Zhu, Zhenzhen Wang

**Affiliations:** a School of Economics and Management, Hunan University of Science and Engineering, Yongzhou, 425199, Hunan, PR China; b School of accounting, Wuhan Qingchuan University, Wuhan, 430204, Hubei, PR China

**Keywords:** Occupational health and safety (OHS), COVID-19, Human factors engineering (HFE), Multiple linear regression (MLR), NetLogo, System dynamics (SD)

## Abstract

Human factors are critical to Occupational Health and Safety (OHS) in construction enterprises. However, comprehensive industry-wide recognition remains challenging, underscoring the need for Human Factors Engineering (HFE) research. This study develops an optimized HFE evaluation model based on fundamental HFE principles. Examining COVID-19's significant impact on construction enterprise OHS, this research employs an empirical investigation of 259 cases, utilizing a model that integrates NetLogo's System Dynamics (SD) and Multiple Linear Regression (MLR) to analyze the interactions between human factors and other variables. The findings reveal four key factors influencing human factors: management, material, environmental, and methodological. These factors demonstrate a quadratic parabolic relationship, with peak influence occurring at step 36 of the research period. Twelve of the 20 survey factors exhibit a linear regression relationship with human factors' four sub-factors, with pre-job training (Q_9_) demonstrating multiple influential interactions. The strongest correlation is between pre-job training (Q_9_) and living materials (Q_14_), with a weight coefficient of .325. Psychological counseling (Q_8_) and living materials (Q_14_) show a close relationship (weight coefficient .301). Notably, Q_9_ and empirical prevention materials (Q_11_) display a negative correlation with a weight coefficient of −.156. This study's practical significance lies in enabling enterprises to identify key HFE control factors and understand critical sub-factors for mitigating COVID-19's adverse impacts.

## 1 Introduction

The global COVID-19 pandemic has severely disrupted the construction industry [[1], [2], [3]], exposing multiple critical risk factors that challenge enterprise management at all organizational levels [4,5]. The pandemic has introduced unprecedented uncertainties to existing risk landscapes [[6], [7], [8]], creating an urgent need for a comprehensive scholarly investigation of Occupational Health and Safety (OHS) factors within the COVID-19 context [9,10]. Emerging research reveals that the global construction industry consistently demonstrates higher accident rates compared to most other sectors [11,12], with particularly pronounced vulnerabilities in developing countries' OHS frameworks [13]. Enhancing OHS effectiveness is critical to safeguarding the well-being of both construction enterprise managers and on-site personnel [14]. Consequently, strategic OHS management demands immediate and sustained organizational attention.

Previous scholarly investigations have employed diverse analytical approaches, including comprehensive OHS influencing factor analyses focused on on-site workers [15] and sophisticated multi-level factorial methodologies [16]. This study aims to design a five-factor scale, design several topics through literature analysis expert investigation, and interview, and complete the empirical investigation [4,17,18].

Human Factors Engineering (HFE)—alternatively termed ergonomics—is a multidisciplinary field examining complex interactions between individuals and their systemic environments, encompassing working conditions, technological tools, and computational interfaces. These interactions affect human behavior and performance. These complex factors, as previously studied by scholars, play an interactive role in many industry fields, such as human cognitive engineering, physics ergonomics, and human-computer interaction. The applied research in the field of HFE provides rich knowledge and a practical foundation for human characteristics and limitations. The fundamental objective of HFE is to strategically design systems that align with human capabilities and accommodate inherent physiological and cognitive constraints [19]. Initially emerging in aviation research [20], HFE subsequently expanded into military applications [21,22] before proliferating across industrial engineering and manufacturing domains, progressively refining human-machine interface optimization [[23], [24], [25]]. In the early 21st century, HFE has experienced exponential growth, expanding beyond traditional engineering domains to encompass diverse sectors including service industries and environmental protection [[26], [27], [28], [29], [30]]. HFE comprehensively examines the intricate interactions between workplace design, environmental conditions, and human physiological and functional characteristics. HFE's primary objective is to optimize worker well-being—encompassing physical, psychological, and occupational health—while simultaneously enhancing workplace productivity [31]. Extensive research demonstrates a critical correlation between human factors, project quality, and workplace environments, evidencing the transformative potential of strategic human intervention in project management [26,32,33]. Consequently, a central aim of this research is to systematically apply Human Factors Engineering principles to OHS management within construction enterprises [[34], [35], [36]].

NetLogo-based System Dynamics (SD) modeling offers a sophisticated analytical approach, enabling comprehensive exploration of interactional dynamics between individual factors and visualization of complex relational processes through dynamic curve representations [[37], [38], [39], [40], [41], [42]]. Grounded in Human Factors Engineering principles, this research employs advanced SD modeling and simulation techniques to investigate the intricate, multidirectional relationships among human factors and associated variables [[43], [44], [45], [46], [47]]. To complement the SD analysis, Multiple Linear Regression (MLR) methodology was applied to rigorously examine the complex interrelationships among research sub-factors [48,49].

This research provides critical insights into pivotal factors influencing construction enterprise operations. By systematically identifying and mitigating risk factors, the study aims to develop strategic interventions that meaningfully address the ongoing challenges posed by the COVID-19 pandemic.

## 2 Methods

### 2.1 Research process design

The research methodology is comprehensively illustrated in Fig. 1, delineating a structured four-stage investigative approach. The initial phase involved a comprehensive literature review and expert consultation to develop a robust survey instrument, incorporating iterative pre-testing and systematic optimization. The second stage focused on systematic questionnaire administration, data collection, and preliminary analytical assessment. The third stage involved constructing a comprehensive SD model using NetLogo, with subsequent curve simulation to visualize complex interactional dynamics. The fourth stage employed MLR techniques to examine the interrelationships among human factors' four sub-components, providing a nuanced statistical exploration. Finally, the analysis result "Result" was obtained.

**Fig. 1:** Process analysis.

### 2.2 Sample dataset design

#### 2.2.1 Data source analysis

The comprehensive questionnaire comprised 27 meticulously designed questions: six demographic items, 20 scaled assessment questions, and one open-ended response section, ensuring a multifaceted data collection approach. Table 1 systematically categorizes the 20 scaled questions across five principal factor domains: Human, Material, Management, Method, and Environmental factors. "Code" referred to the problem code Q_7_∼ Q_26_, and "Initial value" referred to the average value of each variable of the recovered data, which was also the initial value of the flow variables in the SD model. "Description" was the short name of the questions in the questionnaire. The research yielded 259 validated questionnaires, representing a robust and comprehensive data collection effort. For the text of the questionnaire, please see Supplementary A.

**Table 1:** Variable design and description table.

Factor	Code	Initial Value	Description
Personal Information	Q_1_	–	age
	Q_2_	–	educational background
	Q_3_	–	work unit type
	Q_4_	–	position
	Q_5_	–	professional title
	Q_6_	–	How long have you worked?
Human	Q_7_	4.39	self-confidence
	Q_8_	3.98	psychological counseling
	Q_9_	4.51	pre-job training
	Q_10_	4.05	personnel mobility
Material	Q_11_	3.34	epidemic prevention materials
	Q_12_	3.89	fire fighting facilities
	Q_13_	3.76	electrical equipment
	Q_14_	4.46	living materials
Management	Q_15_	3.02	the legal system
	Q_16_	3.96	safety management
	Q_17_	3.41	emergency management
	Q_18_	4.17	residential health
Method	Q_19_	4.18	filing management
	Q_20_	4.22	remote sharing
	Q_21_	3.82	scientific and technological innovation
	Q_22_	4.12	safety control
Environment	Q_23_	4.02	environmental pollution
	Q_24_	4.22	divisional prevention and control
	Q_25_	3.90	healthy buildings
	Q_26_	3.68	fire risk

#### 2.2.2 Data source analysis

As illustrated in Table 2, the survey data were collected through three primary channels: WeChat (71.43 %), mobile submissions, and web links, demonstrating a diverse and accessible data collection strategy.

**Table 2:** Analysis of survey questionnaire sources and channels.

Source channel	Number of questionnaires	Percentage
WeChat	185	71.43 %
Mobile submission	54	20.85 %
Link	20	7.72 %

Total	259	100 %

## 3 Result

### 3.1 Statistical analysis

#### 3.1.1 Indicator description

A total of 259 valid questionnaires were gathered from the survey, with the statistical outcomes displayed in Table 3, titled 'Indicator Description Statistical Table'. The Minimum value was observed to be 1, the Maximum value was 6, the Mean value ranged between 1 and 4, the Mean Standard Error was between .04 and .20, and the Standard Deviation value was within .5–2. Table 3, Table 4 delineate the Q_1_ to Q_6_ indicators for all demographic variables, respectively, to evaluate the validity of the statistical findings.

**Table 3:** Indicator description statistical table.

	N	Minimum	Maximum	Mean		Std. Deviation
	Statistic	Statistic	Statistic	Statistic	Std. Error	Statistic
1. Your age? (Q_1_)	259	1	4	2.51	.062	1.001
2. What is your educational background? (Q_2_)	259	1	4	2.10	.032	.522
3. What is your work unit type? (Q_3_)	259	1	6	2.53	.123	1.973
4. What is your position? (Q_4_)	259	1	3	1.81	.042	.676
5. Your professional title? (Q_5_)	259	1	4	3.05	.052	.836
6. How long have you worked in a construction enterprise? (Q_6_)	259	1	4	3.17	.070	1.122

Valid N (listwise)	259

**Table 4:** Frequency table of Q_1_∼Q_6_.

Valid		Frequency	Percent	Valid Percent	Cumulative Percent
Q_1_	under 30 years old	48	18.5	18.5	18.5
	30–39 years old	80	30.9	30.9	49.4
	40–49 years old	82	31.7	31.7	81.1
	50 years old and above	49	18.9	18.9	100.0
	Total	259	100.0	100.0	
Q_2_	middle school and below	15	5.8	5.8	5.8
	University (undergraduate, junior college)	210	81.1	81.1	86.9
	master	26	10.0	10.0	96.9
	doctor	8	3.1	3.1	100.0
	Total	259	100.0	100.0	
Q_3_	construction unit	148	57.1	57.1	57.1
	supervision unit	6	2.3	2.3	59.5
	developer	22	8.5	8.5	68.0
	universities and research institutions	34	13.1	13.1	81.1
	government	2	.8	.8	81.9
	others	47	18.1	18.1	100.0
	Total	259	100.0	100.0	
Q_4_	company-level (or head office) manager	88	34.0	34.0	34.0
	project department (or branch) manager	132	51.0	51.0	84.9
	team (or worker)	39	15.1	15.1	100.0
	Total	259	100.0	100.0	
Q_5_	senior	12	4.6	4.6	4.6
	vice senior	48	18.5	18.5	23.2
	intermediate	114	44.0	44.0	67.2
	Junior and below	85	32.8	32.8	100.0
	Total	259	100.0	100.0	
Q_6_	less than 2 years	37	14.3	14.3	14.3
	2–5 years	33	12.7	12.7	27.0
	6–9 years	38	14.7	14.7	41.7
	10 years and above	151	58.3	58.3	100.0
	Total	259	100.0	100.0	

As per Table 4, the total proportion of participants aged 30 to 49 in Q1 constituted 62.6 %, representing the majority. The proportion of University attendees (undergraduates, junior college students) in Q2 constituted 81.1 %, signifying the vast majority. The proportion of construction units in Q3 unit sources represented 57.1 %, denoting the majority. The proportion of project department (or branch) managers in Q4 represented 51.0 %, nearly half of the total. The combined proportion of junior and intermediate professional titles in Q5 accounted for 76.8 %, a relatively high fig. 58.3 % of Q6 employees had a work experience of over 10 years, a notably high figure.

#### 3.1.2 Data statistical description

The data in this study were derived from the Likert scale, which is classified as structural data. Therefore, it was essential to conduct an effectiveness and reliability analysis.

(1) Data Validity Analysis

Validity represents the extent to which a measurement tool can accurately measure the attributes it is intended to measure. It is typically categorized into Content validity, Construct validity, and other major types.

1) The Content validity analysis of the questionnaire was partially reliant on the scale that has been extensively used both domestically and internationally, thus yielding good results. The questionnaire is independently developed, and the questionnaire items are summarized through occupational health and safety-related cases of construction enterprises. After conducting preliminary investigations and before finalizing the questionnaire, discussions were held with the interviewees and industry experts, and some incomplete content was revised. This can ensure that the designed questionnaire has good content validity.
2) Due to the large number of variables in the questionnaire design, it is necessary to conduct an exploratory factor analysis on the structural validity of the questionnaire and effectively classify the factors. This study used SPSS23.0 software for principal component analysis and grouped the influencing factors. Exploratory factor analysis was conducted on both grouped factors and overall factors. Moreover, the KMO (Kaiser Meyer Olkin) test and Bartlett's sphericity test were conducted before factor analysis to determine whether variables are suitable for factor analysis. Usually, KMO statistical data has corresponding standards, and values above .90 are usually the best, while values below .50 are unacceptable. Moreover, from Table 5, it can be seen that the test results of this study show that the KMO sample detection values of each scale are all greater than .7 (measured value is. 912, which is an excellent level), and the Bartlett sphere test values are all less than .001, indicating good effectiveness of factor analysis.

**Table 5:** KMO and Bartlett's test.

Kaiser-Meyer-Olkin Measure of Sampling Adequacy.		.912
Bartlett's Test of Sphericity	Approx. Chi-Square	2400.469
	df	190
	Sig.	.000

From the above KMO statistics, it can be concluded that all measurement items in the questionnaire are reasonably and effectively distributed across several potential common factors, and the factor loadings of all measurement items are greater than .5, while the factor loadings of other potential variables are less than .5. Therefore, the convergent validity and discriminant validity of the collected questionnaire data are both good. By removing factors with a factor load less than .5 and their effects, the final effective results of exploratory factor analysis can be obtained. Overall, the collected questionnaire data has good convergence and differential validity.

(2) Data Reliability Analysis

Finally, after conducting exploratory factor analysis as described above, statistical analysis tools and Cronbach's alpha coefficients were used again to determine whether the designed scale had a high degree of internal consistency. The standard usually stipulates that α ≥ 0.7 is considered high reliability, and α ≤ 0.35 is considered low reliability. The results of this inspection are shown in Table 6. Due to the Cronbach's alpha coefficients of all factors being greater than .6, this indicates that the reliability of the collected questionnaire data is high and can be used for subsequent analysis and simulation.

**Table 6:** Reliability statistics.

Cronbach's Alpha	Cronbach's Alpha Based on Standardized Items	N of Items
.913	.918	20

Therefore, based on the above-assumed model and analysis results, the causal model of human factors can be considered effective and reliable. Combined with practical background, this model has significant practical application significance.

### 3.2 SD Based on NetLogo

In conjunction with the principles of HFE, the SD model was designed based on the NetLogo platform to investigate the impact process and degree of the other four types of factors on Human factors (refer to Fig. 2). It could be seen from this figure that Humans had four rheological quantities Q7∼Q10, corresponding to Table 1 of Q_7_∼ Q_10_, and the initial value of flow variable Q7 was 4.39. The initial values of other flow variables were also from Table 1 corresponding initial value. E1 was a constant with a value of 100, which referred to the limit value of the stock variable Human. R1 was the flow rate variable. Similarly, refer to Table 1 to understand the meanings of variables and constants corresponding to other factors. Some procedures and formulas (Formula 1) in the SD flow diagram were as follows:

**Fig. 2:** Sd based on NetLogo.

Report value of flow.

to-report R1

report (ln((E1 - Human)/(Q7 + Q8 + Q9 + Q10 + .25 ∗ (Material + Management + Method + Environment)))

) ∗ dt.

End.

For the complete program source code, please see Supplementary B.

(Formula 1) $$\begin{array}{l} \ln(\left(E1-Human\right)/(Q7+Q8+Q9+Q10+0.25*\\ \left(Material+Management+Method+Envirenment\right))) \end{array}$$

### 3.3 Plot of SD

Currently, the designed SD flowchart program is running on the NetLogo platform. Fig. 3 displays the dynamic curve, outputting the SD diagram concerning Human factors. It could be seen that the Human curve was a quadratic parabola, and gradually reached the peak in the first 36 steps, and then gradually decreased, which indicated that Human factors were most affected by the superposition of the other four types of factors in the previous 36 steps of the study period. It could also be seen that the other four types of factors were exponential curves. In step 72, there was a rapid increase to a gradual increase. At the same time, the "Impact_Value" of the influence curve of the four types of factors were manufacturing, material, environment, and method from top to bottom. It could be seen that management had the greatest impact on Human factors, and other factors affect Human factors at one time.

**Fig. 3:** Plot of SD

### 3.4 MLR analysis

#### 3.4.1 Regression equation design

To delve deeper into the relationship between the sub-factors Q_7_∼Q_10_ of human factors and other sub-factors, a stepwise MLR method was employed to construct the corresponding model. Firstly, Q_7_ was used as an example for stepwise regression analysis, and the analysis results were shown in Table 7, Table 8, Table 9. The goodness of fit R Square in step 4 of Table 7 was .344, and Adjusted R Square was .334, and the Durbin-Watson value was 2.055, indicating a good fitting effect. In the total regression equation (see Table 8), the significance of the F test sig was .016, and the result was significant.

**Table 7:** Model summary^b^ of Q_7_.

Model	R	R Square	Adjusted R Square	Std. Error of the Estimate	Change Statistics					Durbin-Watson
					R Square Change	F Change	df1	df2	Sig. F Change	
1	.473^a^	.224	.220	.986	.224	73.975	1	257	.000	
2	.544^b^	.296	.291	.941	.073	26.512	1	256	.000	
3	.573^c^	.329	.321	.920	.032	12.331	1	255	.001	
4	.587^d^	.344	.334	.912	.015	5.898	1	254	.016	2.055

a Predictors: (Constant), 14. [remote sharing], 6. [fire fighting facilities], 12. [residential health], 19. [healthy buildings].

b Dependent Variable: 1. [self-confidence].

**Table 8:** ANOVA^a^ of Q_7_.

Model		Sum of Squares	df	Mean Square	F	Sig.
1	Regression	71.931	1	71.931	73.975	.000^b^
	Residual	249.899	257	.972		
	Total	321.830	258			
2	Regression	95.382	2	47.691	53.915	.000^c^
	Residual	226.448	256	.885		
	Total	321.830	258			
3	Regression	105.828	3	35.276	41.645	.000^d^
	Residual	216.002	255	.847		
	Total	321.830	258			
4	Regression	110.729	4	27.682	33.308	.000^a^
	Residual	211.101	254	.831		
	Total	321.830	258			

a Predictors: (Constant), 14. [remote sharing], 6. [fire fighting facilities], 12. [residential health], 19. [healthy buildings].

**Table 9:** Coefficients^a^ of Q_7_.

Model		Unstandardized Coefficients		Standardized Coefficients	t	Sig.	Collinearity Statistics	
		B	Std. Error	Beta			Tolerance	VIF
4	(Constant)	1.318	.276		4.769	.000		
	14. [remote sharing]	.242	.070	.225	3.463	.001	.614	1.629
	6. [fire fighting facilities]	.175	.048	.208	3.676	.000	.806	1.240
	12. [residential health]	.190	.070	.178	2.715	.007	.604	1.655
	19. [healthy buildings]	.149	.061	.158	2.429	.016	.612	1.634

a Dependent Variable: 1. [self-confidence].

In this stepwise regression analysis, all sub-factors within the five types of factors were initially regressed with Q_7_, yielding the regression coefficient table displayed in Table 9. From this table, it could be seen that the VIF values were less than 2, which could be determined that there was no Multicollinearity relationship between the factors. A significant regression relationship was observed between the dependent variable self-confidence and the four independent variables, namely fire lighting facilities (Q_12_), residential health (Q_18_), remote sharing (Q_20_), and health buildings (Q_25_) (refer to Table 1, Table 9). Therefore, the constructed MLR equation was Equation (1).

Similarly, corresponding regression analyses were conducted on Q_8_, Q_9_, and Q_10_, resulting in the construction of standardized regression equations Equation (2), Equation (3), and Equation (4).

From the regression coefficients of factors Q_7_, Q_8_, Q_9_, and Q_10_, in Table 9, Table 10, Table 11, Table 12, it can be seen that the t-values, p-values, or standard errors of all factor variables are within the valid range. Therefore, the constructed regression equations are all effective and reliable.

(Equation 1) $$Q_{7}=0.208Q_{12}+0.178Q_{18}+0.225Q_{20}+0.158Q_{25}$$

(Equation 2) $$Q_{8}=0.286Q_{12}+0.301Q_{14}+0.197Q_{15}+0.169Q_{20}$$

(Equation 3) $$Q_{9}=-0.156Q_{11}+0.169Q_{12}+0.325Q_{14}+0.163Q_{16}+0.243Q_{19}+0.122Q_{21}$$

(Equation 4) $$Q_{10}=0.149Q_{11}+0.228Q_{17}+0.225Q_{19}+0.217Q_{22}$$

**Table 10:** Coefficients^a^ of Q_8_.

Model		Unstandardized Coefficients		Standardized Coefficients	t	Sig.	Collinearity Statistics	
		B	Std. Error	Beta			Tolerance	VIF
4	(Constant)	−.290	.321		−.901	.368		
	8. [living materials]	.409	.076	.301	5.373	.000	.702	1.425
	6. [fire fighting facilities]	.272	.049	.286	5.512	.000	.816	1.226
	9. [the legal system]	.174	.044	.194	3.969	.000	.920	1.087
	14. [remote sharing]	.206	.068	.169	3.043	.003	.714	1.400

a Dependent Variable: 2. [psychological counseling].

**Table 11:** Coefficients^a^ of Q_9_.

Model		Unstandardized Coefficients		Standardized Coefficients	t	Sig.	Collinearity Statistics	
		B	Std. Error	Beta			Tolerance	VIF
6	(Constant)	.987	.241		4.097	.000		
	8. [living materials]	.348	.059	.325	5.911	.000	.637	1.570
	13. [filing management]	.210	.050	.243	4.211	.000	.579	1.726
	10. [safety management]	.156	.049	.163	3.189	.002	.732	1.365
	6. [fire fighting facilities]	.126	.040	.169	3.160	.002	.675	1.481
	5. [epidemic prevention materials]	−.115	.036	−.156	−3.239	.001	.829	1.206
	15. [scientific and technological innovation]	.096	.044	.122	2.178	.030	.611	1.638

a Dependent Variable: 3. [pre-job training].

**Table 12:** Coefficients^a^ of Q_10_.

Model		Unstandardized Coefficients		Standardized Coefficients	t	Sig.	Collinearity Statistics	
		B	Std. Error	Beta			Tolerance	VIF
4	(Constant)	1.021	.305		3.352	.001		
	16. [safety control]	.234	.063	.217	3.696	.000	.799	1.252
	11. [emergency management]	.204	.052	.228	3.948	.000	.826	1.211
	13. [filing management]	.226	.057	.225	3.982	.000	.868	1.152
	5. [epidemic prevention materials]	.128	.049	.149	2.632	.009	.863	1.159

a Dependent Variable: 4. [personnel mobility].

From Equation (1), it is evident that an MLR relationship exists between Q_7_ and Q_12_, Q_18_, Q_20_, and Q_25_. In other words, the sub-factor Q_7_ in human factors has the closest association with sub-factors Q_12_, Q_18_, Q_20_, and Q_25_, indicating an MLR relationship.

Similarly, the sub-factor Q_8_ in human factors had the closest relationship with sub-factors Q_12_, Q_14_, Q_15_, and Q_20_, and there was an MLR relationship. The relationship between sub-factor Q_9_ and sub-factors Q_11_, Q_12_, Q_14_, Q_16_, Q_19_, and Q_21_ was the closest, and there was an MLR relationship. The relationship between sub-factor Q_10_ and sub-factors Q_11_, Q_17_, Q_19_, and Q_22_ was the closest, and there was an MLR relationship.

In summary, Q_9_ was a person whose sub-factors were influenced by other sub-factors. Q_13_, Q_23_, Q_24_, and Q_26_ did not feature in the regression equation, necessitating separate analysis of these four sub-factors.

#### 3.4.2 Regression coefficient relationship diagram

To intuitively reflect the regression relationship between the sub-factors of human factors and other sub-factors, the corresponding sub-factor numbers such as Q_7_ correspond to a circle of 7, and other sub-factors were similar to the corresponding numbers. At the same time, the coefficients were used as weight labels on the cutting line (see Fig. 4). The circle in the middle row of this figure was divided into Material (11, 12, 14), Management (15–18), Method (19–22), and Environment (25) based on four types of factors.

**Fig. 4:** Regression coefficient relationship diagram.

As shown in Fig. 4, the impact weight between factors 9 and 11 was negative (−.156), indicating that pre-job training could greatly reduce the risk of epidemic prevention. The maximum impact weight (weight coefficient of .325) was between factors 9 and 14, and there was a positive correlation between daily necessities and pre-job training. Secondly, factors 8 and 14 exerted a significant influence on the weight, with a weight coefficient value of .301, indicating a significant positive correlation between them. In addition, 13,23,24,26 did not enter the regression relationship diagram, and the meanings of these four numbers were electrical equipment, environmental pollution, visual prevention and control, and fire risk. Given that these four sub-factors are expected to significantly impact human factors, they warrant special attention.

## 4 Discussion

Recent years have seen the application of HFE studies in the medical field, primarily focusing on enhancing aspects of the human body, psychology, and equipment [[50], [51], [52], [53]]. HFE research in construction engineering has been relatively scant, particularly concerning the impact of diverse factors on human elements [[54], [55], [56], [57]]. Based on previous studies, this study put forward the analysis of the influence of Human factors on HFE through empirical investigation. Given the multitude of factors influencing Human elements, this study primarily utilized four types of factors recognized by scholars: material, management, environmental, and method factors. These were used to construct a simulation model, subsequently investigating the relationships between sub-factors and formulating a regression equation [[58], [59], [60]].

Many factors affect OHS, especially for construction enterprises that belong to high-risk industries [[61], [62], [63]]. Choosing OHS in construction enterprises and exploring the human factors engineering influencing factors of such enterprises has significant practical significance [[64], [65], [66]]. The study's findings also suggest that certain influencing factors can be viewed as key focal points, offering guidance for managing human factors engineering within enterprises.

This study primarily innovated in two aspects. First, combined with the principles of HFE, an SD simulation model based on NetLogo was built to simulate and showed the influence process and degree of the other four types of factors that affect Human factors. The second was to further analyze the regression relationship between the four sub-factors in human factors and other sub-factors based on the analysis of categorical factors, and construct a regression relationship graph, capturing the main controlling sub-factors.

This study primarily took into account the following essential steps. The first was the design of the survey scale. Using the Likert five-level scale, 20 scale questions were designed. At the same time, 6 classification questions were designed for the personal information of construction enterprises. However, this study did not analyze the 6 items of personal basic questions. Secondly, the NetLogo platform was commonly used in social sciences was used to build the influence model of five categories of factors in combination with the application of SD. Finally, the MLR relationship among the sub-factors was deeply analyzed, and the regression equation of the four sub-factors of Human factors was constructed. This not only showed the dynamic relationship and development trend of the five factors from the macro level but also revealed the influence relationship between the sub-factors from the micro-level. It could be seen that this study revealed the influence relationship between various factors at all levels from macro to micro, from major factors to sub-factors. This was the highlight of this study.

The primary limitation of this study was that the sample size of the recovered data was 259, roughly ten times the number of questions (26). Subsequent research plans to augment the sample size to approximately twentyfold. Moreover, the influencing factors and sub-factors of Human elements in HFE may differ across various environments and regions. Thus, accurately and judiciously selecting each factor also presents a challenging issue warranting further exploration.

## 5 Conclusion

Utilizing the principles of HFE and empirical investigation, this study initially employed SD modeling and simulation on the NetLogo platform to procure the simulation curve. It then built an MLR equation for the four sub-factors of Human elements and validated and analyzed the relationship among the sub-factors in the regression equation. The following conclusions were subsequently derived.

Firstly, Human elements were influenced by management, material, environmental, and method factors, and the model, which combined HFE, SD, and MLR, proved to be effective and applicable.

Secondly, Human elements within HFE were holistically affected by the other four types of factors, with the influence curve demonstrating a quadratic parabola relationship. Before 36 steps in the study period, the influence curve gradually rose to the peak, and then slowly declined. The importance of each factor on Human factors was as follows: management factor, material factor, environmental factor, and method factor, and these four factors showed an exponential development trend, with a turning point in the 72 steps of the research period. Consequently, management factors had the most significant impact on Human elements, with steps 36 and 72 representing the crucial control time nodes of HFE throughout the research period.

Thirdly, the MLR equations for each of the four sub-factors in Human elements were valid. Pre-job training (Q_9_) had the highest number of influencing sub-factors (six), which served as the primary controlling sub-factors. Moreover, the weight coefficients of the sub-factor of daily necessities (Q_14_) were relatively large compared to Q_9_ and Q_8_, so special attention should be paid to the sub-factor of Q_14_. In addition, there were a total of 12 sub-factors entering the regression equation, which were factors that human factors engineering needs to pay attention to.

The practical implication of this study lies in aiding construction enterprises to reinforce the control of HFE factors in OHS management amid the COVID-19 environment, thereby mitigating the negative impacts of COVID-19 on OHS management within these enterprises.

From the viewpoint of specific policy applications, construction enterprises should integrate the principles of human factors engineering into their everyday management practices, particularly in the management of production sites, to minimize risks and damages caused by human factors and other factors. Strengthen early management throughout the entire lifecycle of each project. Emphasis should be placed on controlling pre-job training, daily necessities, and other factors among all risk factors. These factors are the key factors in the OHS management of construction enterprises during and after the COVID-19 epidemic, and government departments can take intervention and policy formulation on this basis.

## CRediT authorship contribution statement

**Zhonghong Cao:** Writing – original draft, Validation, Supervision, Software, Resources, Project administration, Methodology, Funding acquisition, Conceptualization. **Junjie Zhu:** Writing – review & editing, Visualization, Software, Resources, Methodology, Investigation, Formal analysis, Data curation. **Zhenzhen Wang:** Writing – review & editing, Validation, Software, Investigation, Data curation.

## Data availability statement

All data, models, and code generated or used during the study appear in the submitted article.

## Ethics statement

The studies involving participants were reviewed and approved by the Research Ethics Committee of Hunan University of Science and Engineering (approval no. XSP2023GLC113), the author ensured that the work described has been carried out by the Code of Ethics of the World Medical Association (Declaration of Helsinki) for experiments involving humans. The participants provided written informed consent to participate in this study.

## Funding

This study was funded by the 2023 Hunan Social Science Achievement Evaluation Committee Project (XSP2023GLC113), the Research Achievements in the Stage of Education Science Planning in Hunan Province, Research on the Path of Occupational Health and Safety Education for College Students under the Overall National Security Concept (XJK23BGD042), and the University level project of Hunan University of Science and Engineering (2022028), and the Key Project of Hubei Provincial Education Science Plan for 2023(2023GA084), and the 2024 Hunan Province Undergraduate Teaching Reform Research Project (202401001394), and the 2024 Hunan Provincial Department of Education Scientific Research Project (24A0596).

## Declaration of competing interest

The authors declare that they have no known competing financial interests or personal relationships that could have appeared to influence the work reported in this paper.
